RETRACTED

# Insight into the Protective Effect of Salidroside against H_2_O_2_-Induced Injury in H9C2 Cells

**DOI:** 10.1155/2021/1060271

**Published:** 2021-11-30

**Authors:** Hui Gao, Xueping Liu, Kunming Tian, Yichong Meng, Cuicui Yu, Yingfu Peng

**Affiliations:** ^1^Department of Pharmacology, School of Medicine, Shaoxing University, Shaoxing 312000, China; ^2^Department of Pharmacology, School of Medicine, Jishou University, Jishou 416000, China; ^3^Department of Pharmacology, School of Medicine, Guangxi University of Science and Technology, Liuzhou 545006, China; ^4^Department of Environmental Toxicity, Zunyi Medical University, Zunyi 563006, China; ^5^Tibet Agricultural Science and Technology Innovation Park, Lhasa, 850000 Tibet, China

## Abstract

Salidroside is the important active ingredient of *Rhodiola* species, which shows a wide range of pharmacological activities such as antioxidative stress, anti-inflammation, and antiliver fibrosis. In this paper, we aimed to study the protective effect and mechanism of salidroside against H_2_O_2_-induced oxidative damage in H9C2 cells by determining cell proliferation rate, intracellular reactive oxygen species (ROS) level, antioxidant enzyme activities, and the expression of apoptosis-related proteins. The results showed that salidroside significantly alleviated cell growth inhibition induced by H_2_O_2_ treatment in H9C2 cells, decreased the levels of intracellular ROS and malondialdehyde (MDA), and increased the activity of superoxide dismutase (SOD) and catalase (CAT); meanwhile, salidroside upregulated the expression of Bcl-2 while downregulated the expression of Bax, p53, and caspase-3 in H_2_O_2_-treated H9C2 cells. Furthermore, the antiapoptotic effect of salidroside was almost eliminated by the knockdown of Bcl-2. In the further exploration, the Bcl-2 expression was decreased by the p53 overexpression and increased by p53 knockdown in H_2_O_2_-treated H9C2 cells. Consequently, salidroside could protect H9C2 cells against H_2_O_2_-induced oxidative damage, and the underlying mechanism may be related to scavenging intracellular ROS, increasing the activities of intracellular antioxidant enzymes and inhibiting the expression of apoptosis-related proteins.

## 1. Introduction

Reactive oxygen species (ROS) is considered as the second messenger in cells, which implicates in the processes of cell proliferation, differentiation, and apoptosis [1]. Researchers have found that ROS-mediated oxidative stress is a key pathophysiological process in myocardial ischemia/reperfusion injury, cardiac hypertrophy, and heart failure [2]. Although hydrogen peroxide (H_2_O_2_) is necessary for normal cell physiology, the overproduction can cause oxidative stress and lead to cellular damage and apoptotic cell death. Recently, a large number of publications have shown that oxidative stress-induced cardiomyocyte apoptosis plays an important role in the development and progression of cardiovascular diseases [3–6]. In this case, the search for new natural compounds which exert effects on inhibiting oxidative stress and reducing cardiomyocyte apoptosis is considered a promising strategy for the improvement of cardiovascular disease. Many natural ingredients such as flavonoids [7, 8], polyphenols [9, 10], and alkaloids [11] have been reported to have antioxidant or protective properties, and they may be valuable for the treatment of myocardial injury.

RETRACTED

Salidroside, a kind of phenolic glycoside compound, is extracted from *Rhodiola* species such as *Rhodiola rosea*, *Rhodiola sachalinensis*, and *Rhodiola crenulata* [12] and possesses the pharmacological effects on antioxidative stress, antidiabetes, anti-inflammation, antiliver fibrosis, and others [13]. In addition, salidroside has shown protective effects in heart diseases such as LPS-induced myocardial injury [14], ischemia-reperfusion myocardial injury [15], doxorubicin-induced cardiac dysfunction [16], and hypoxia-induced myocardial injury [12, 17]. However, oxidative stress is a common phenomenon in heart diseases. For example, the activation of sympathetic nerves and renin angiotensin system can induce the production of a large amount of ROS and promote the development and progress of cardiac hypertrophy by contributing to the disorder of energy metabolism and left ventricular systolic dysfunction [2]. In particular, excessive ROS induce cardiomyocyte apoptosis and then lead to abnormal cardiomyocyte death, which may be one of the important reasons why cardiac hypertrophy progresses to heart failure [2]. Although salidroside exhibits the protective effect against oxidative stress [18, 19], the mechanisms remain unclear. In this research, H9C2 cells derived from embryonic rat heart tissue were exposed to H_2_O_2_ in vitro to establish a cell injury model. The effects of salidroside on the H_2_O_2_-induced damage in H9C2 cells were assessed. The cell viability, morphological changes, apoptosis, and change of antioxidant enzyme content were determined.

## 2. Materials and Methods

### 2.1. Chemicals and Reagents

Salidroside used in this study was purchased from Sigma-Aldrich, China, and the purity was over 99%; 6-carboxy-2′,7′-dichlorofluorescein diacetate (DCF-DA) was purchased from Beijing Solarbio Science Technology (Beijing, China); the assay kits of superoxide dismutase (SOD), catalase (CAT), and malondialdehyde (MDA) were purchased from Nanjing Jiancheng Bioengineering Institute (Nanjing, China). Bcl-2 rabbit polyclonal antibody (D160117), Bax rabbit polyclonal antibody (D220073), cleaved caspase-3 rabbit polyclonal antibody (D164390), and p53 mouse monoclonal antibody (D191060) were purchased from Biotech Bioengineering (Shanghai, China). Phosphorylated NF-*κ*B p65 (p-p65, Ser536) rabbit monoclonal antibody (3033), phosphorylated signal transducer, and activator of transcription 3 (p-STAT3, Tyr705) rabbit monoclonal antibody (9145), and PTEN rabbit monoclonal antibody (9188) were purchased from Cell Signaling Technology (CST, Danvers, MA, USA).

RETRACTED

### 2.2. Cell Culture and Transfection

H9C2 cells were obtained from the Type Culture Collection of the Chinese Academy of Sciences (Shanghai, China) and were cultured in Dulbecco's Modified Eagle's Medium (DMEM, Gibco, NY, USA) supplemented with 10% fetal bovine serum, at 37°C in a humidified atmosphere containing 5% CO_2_.

SiRNA targeting p53 [20] and Bcl-2 [21] were obtained from GenePharma (Shanghai, China). H9C2 cells were seeded in 12-well plates at a density of 1 × 10^5^ cells/well for 48 h, and the transfection was operated until cells reached to 60-80% confluence. The cells were then transfected with siRNA targeting p53 or Bcl-2 using Lipofectamine 3000™ reagent according to the manufacturer's instructions, and nontargeting siRNA was used as a negative control (NC).

### 2.3. Cell Viability

Cell proliferation was evaluated by the MTT assay. Firstly, cells were plated at a density of 1 × 10^5^ cells/well in 12-well plate overnight. Then, pretreated with salidroside (0, 25, 50, 100, 200, 400 *μ*M) for 1 h and cotreated with hydrogen peroxide (H_2_O_2_) (0, 50, 100, 200, 400, 800 *μ*M) for 24 h, MTT working solution (Promega, Madison, WI, USA) was added to the culture plates for 4 h at 37°C. The absorbance at 450 nm was measured. The results were expressed as a percentage of the control, considered as 100%.

### 2.4. Apoptosis Assay

Apoptotic cells were detected with an In Situ Cell Death Detection Kit (Thermo Fisher, Waltham, MA, USA; Catalog No. C1024) according to the manufacturer's protocol. Briefly, cells were fixed with 4% paraformaldehyde for 15 min at 37°C. Blocking buffer (3% of H_2_O_2_ in methanol) was added to the wells, and then cells were permeabilized with 0.1% Triton X-100 for 2 min on ice. The cells were incubated with TUNEL reaction mixture for 1 h at 37°C. 4′,6-diamidino-2-phenylindole (DAPI, Sigma-Aldrich, St. Louis, MO, USA) was used to counterstain the nuclei, and the numbers of TUNEL-positive cells were recorded.

### 2.5. Identification of Intercellular ROS Level

Intracellular ROS was detected using DCFH-DA (Beyotime, Shanghai, China), a fluorescent dye sensitive to oxidation, according to the previous study [7]. In brief, the cells were incubated in serum-free DMEM with 10 *μ*M of DCFH-DA for 20 min and then were washed with PBS three times. The fluorescence was detected by the microplate reader, the excitation of which was set at 488 nm, and the emission at 525 nm. The percentage of the control was adopted to express the intracellular ROS.

RETRACTED

### 2.6. Determination of the Activity of SOD and CAT and the Level of MDA

H9C2 cells in a six-well plate were washed twice with cold PBS and then lysed with RIPA buffer. The enzyme activities of SOD and CAT and the level of MDA were determined, according to the manufacturer's protocols from Jiancheng Biological Engineering Institute (Nanjing, China).

### 2.7. The Flow Cytometric Apoptosis Analysis

The death of cells was analyzed using the Annexin V-FITC/PI double staining kit (Sigma-Aldrich, USA). H9C2 cells (1 × 10^6^ cells/well) were collected and rinsed twice using cold PBS and then incubated in the Annexin V/PI labeling reagent for 20 min at room temperature in darkness. The cell cycles were detected by flow cytometry (FACSCanto II Analyzer, BD, USA).

### 2.8. Western Blotting Assay

H9C2 cells were collected and then lysed using RIPA. The protein concentrations were determined using a BCA Protein Assay Kit (Beyotime, Shanghai, China). Protein (20 *μ*g) was separated in 10% SDS-PAGE and then transferred to PVDF membranes. After that, the membranes were blocked in Tris-buffered saline/Tween 20 (TBST) with 5% defatted milk for 1 h at room temperature and then incubated with primary antibodies overnight at 4°C and secondary antibodies for 1 h at room temperature. The bands were developed with an enhanced chemiluminescence substrate and detected by the ChemiScope mini (Clinx Science Instruments, Shanghai, China). The intensities of the blots were quantified with Image J V1.8 (National Institutes of Health, Bethesda, MD, USA).

### 2.9. Statistical Analysis

The measurement data were expressed as mean ± standard deviation. Statistical analysis was performed with analysis of variance (ANOVA) followed by Bonferroni posthoc test using SPSS 23.0 (IBM, San Francisco, CA, USA). *p* < 0.05 was considered statistically significant.

## 3. Results

### 3.1. Salidroside Alleviated the Decreased Cell Viability and the Increased ROS Level in H_2_O_2_-Treated H9C2 Cells

The cell viability was determined by the MTT assay to evaluate the cytotoxic effects of salidroside on H9C2 cells. The amount of 100 *μ*M of salidroside was confirmed as nontoxic concentration (Figure 1(a)). In addition, the results revealed that with the increase of H_2_O_2_ concentration, the cell viability of H9C2 was decreased.400 *μ*M of H_2_O_2_ was used to induce oxidativestress in H9C2 cells as the cell viability was reduced to 51% at the concentration (Figure 1(b)). Compared with H_2_O_2_ treatment, the cell viability in 100 *μ*M of salidroside-treated H9C2 cells was significantly increased to 85% (Figure 1(c)). Furthermore, H_2_O_2_ treatment could also significantly induce the increase of intracellular ROS level in H9C2 cells, while the ROS level was significantly reduced by salidroside treatment in a dose-dependent manner (Figure 1(d)). These results indicated that salidroside can improve oxidative stress injury induced by H_2_O_2_ in H9C2 cells.

RETRACTED

### 3.2. Salidroside Recovered the Decreased Enzyme Activities of SOD and CAT and Decelerated the Elevated Level of MDA

It is well known that SOD and CAT, which act as endogenous antioxidative enzymes, protect cells from ROS-induced injury (Figure 2(a)) [22, 23]. MDA, a lipid peroxidation product, is usually used to assess the level of lipid peroxidation [23]. As shown in Figures 2(b) and 2(c), H9C2 cells were pretreated with salidroside (25, 50, and 100 *μ*M) for 24 h and then coincubated with H_2_O_2_ for another 4 h, and the activities of SOD and CAT were increased by salidroside pretreatment in a dose-dependent manner, respectively, when compared with H_2_O_2_ treatment. On the contrary, intracellular MDA level was reduced by salidroside pretreatment in a dose-dependent manner (Figure 2(d)).

### 3.3. Salidroside Inhibited the Apoptosis Induced by H_2_O_2_

Bcl-2 and Bax are two well-known proteins in the Bcl family, which are closely linked to an imbalance in the mitochondrial homeostasis [24]. As shown in Figure 3, H_2_O_2_ treatment resulted in a decrease of the expression of antiapoptotic protein Bcl-2 and the increase of the proapoptotic protein Bax in dose-dependent manner. On the contrary, salidroside reverses the situation in a dose-dependent manner. In addition, the expression of cleaved caspase-3 was decreased in H9C2 cells pretreated with salidroside and then incubated with H_2_O_2_ when compared with H_2_O_2_ treatment alone (Figure 3).

Salidroside might elevate the expression of Bcl-2 to alleviate oxidative injury by H_2_O_2_ as Bcl-2 is a negative upstream regulator of both Bax and caspase-3 [25]. Thus, the expression of Bcl-2 was knocked down to verify the assumptions. First, the expression of Bcl-2 protein was knocked down by siRNA targeting Bcl-2 to 36% of the control (Figure 4(a)). As expected, the reduction of the expression of Bax and active caspase-3 due to salidroside treatment was impaired by the knockdown of Bcl-2 in H_2_O_2_-stimulated cells (Figure 4(b)). Furthermore, H_2_O_2_ treatment also resulted in the increase of nuclear pyknosis and fragmentation when tested by Hoechst staining, which was inhibited by salidroside treatment, but this effect of salidroside was impaired by the knockdown of Bcl-2 (Figure 4(c)). These results indicated that the upregulation of the Bcl-2 expression was associated with the antiapoptotic effect of salidroside in H_2_O_2_-induced apoptosis. The hypothesis was further confirmed by flow cytometry analysis (Figure 4(d)).

RETRACTED

### 3.4. The Inhibition of p53 Was Involved in the Protective Effect of Salidroside in H_2_O_2_-Induced Apoptosis

It was still unclear that how Bcl-2 expression was elevated by salidroside. The upstream regulators of Bcl-2 mainly include p53, STAT3, NF-*κ*B p65, and PTEN [25]. The phosphorylation of STAT3 at Tyr705 site means the increase of transcriptional activity, which is regarded as a marker of activation. The same is true for NF-*κ*B p65 at Ser536 site. As shown in Figure 5, compared with H_2_O_2_ treatment, the protein expressions of p53, p-STAT3, and p-p65 were significantly decreased after salidroside intervention, whereas the protein expression levels of PTEN were not changed much.

The inhibition of NF-*κ*B p65 and STAT3 might not be involved in the upregulation of the Bcl-2 expression by salidroside because their activation can induce the increase of the Bcl-2 expression [25]. In addition, PTEN, an inhibitor of Bcl-2 [25], was not changed by salidroside. Thus, the downregulation of p53 expression might relate to the increased expression of Bcl-2 in salidroside-treated cells. The relationship between p53 and Bcl-2 needs to be confirmed clearly in the following operation. As shown in Figure 6(a), the expression of Bcl-2 was reduced but the expression of Bax was increased by the overexpression of p53. On the contrary, the downregulation of the Bcl-2 expression and the up-regulation of the Bax expression were reversed by the knockdown of p53 when compared with H_2_O_2_ treatment (Figure 6(b) and 6(c)). These results indicated that the increase of the expression of Bcl-2 and the reduction of the expression of Bax induced by the inhibiting the effect of p53 were involved in the protective effects of salidroside in H_2_O_2_-induced injury in H9C2 cells.

## 4. Discussions

SOD and CAT are important antioxidant enzymes in cells and act as an important components against oxidative stress, effectively eliminating ROS, preventing lipid peroxidation, and improving the antioxidant capacity of the body [26]. MDA is the final decomposition product of lipid peroxidation, and its content is an important indicator of the levels of reactive lipid peroxides and reactive oxygen radicals [27]. The excessive production and accumulation of ROS could result in lipid peroxidation of cell membranes, which eventually cause oxidative damage or apoptosis [28]. H_2_O_2_ is a crucial product in the oxidative response and commonly used as an inducer of oxidative damage in vitro, which can activate the mitochondrial apoptosis pathway and then lead to the decreased cell survival [2]. Our results showed that salidroside can significantly increase SOD and CAT activities, effectively inhibit the formation of ROS, and reduce MDA content in H_2_O_2_-treated H9C2 cells obviously (Figure 2). H9C2 cells were protected from H_2_O_2_-induced oxidative damage depending on the protective effect of salidroside. It was clearly suggested that salidroside could act as an activator with antioxidative properties. The endogenous antioxidant defense system by increasing the activities of intracellular antioxidant enzymes was also strengthened. Other researchers also found that salidroside upregulated the activities of antioxidative enzymes such as SOD, CAT, and glutathione peroxidase and reduced the content of MDA in rat livers [29–31]. In addition, salidroside has multiple alcoholic hydroxyl groups and one phenolic hydroxyl group (Figure 2(a)), which might capture unpaired electrons to scavenge free radicals, thereby protects cells from oxidative stress. However, the ability of salidroside in eliminating free radicals cannot be deduced in the current study.

RETRACTED

Heart failure is the common terminal stage of a variety of heart diseases, in which the loss of cardiomyocytes plays an important role. Apoptosis caused by oxidative damage seems to be the predominant pathway in this process [24]. There are numerous events associated with apoptosis mediated by apoptotic proteins. Therefore, we investigated the effect of salidroside on protein expressions of Bcl-2 and Bax in cells stimulated by H_2_O_2_. Bcl-2 can bind to Bax and other proapoptotic proteins, and the ratio of Bcl-2/Bax is critical for whether apoptosis occurs [32]. H_2_O_2_ treatment exerted opposite effects on these two apoptotic related proteins. As shown in Figure 3, the expression of antiapoptotic protein Bcl-2 was decreased, while Bax expression (proapoptotic protein) was increased, both of which are closely linked to an imbalance in the mitochondrial homeostasis. In general, the decline of Bcl-2/Bax ratio induces cell apoptosis through activating caspase-3, a final executor of apoptosis [33]. The active caspase-3 enters the nucleus to activate the endonuclease, which causes DNA cleavage and leads to cell apoptosis [34]. In the present study, we observed that the treatment with salidroside significantly upregulated the protein expression of Bcl-2 and simultaneously downregulated the protein expression of Bax and cleaved caspase-3 when compared with H_2_O_2_ treatment (Figure 3). Furthermore, the effects of salidroside on these protein expressions were almost eliminated by the knockdown of Bcl-2. The antiapoptotic effect of salidroside was also confirmed by the morphological changes of apoptotic cells observed by Hochest staining and Annexin V/PI assay (Figure 4(d)). Taken together, these results suggested that the cardioprotective effect of salidroside was related to increasing the expression of Bcl-2 and thereby inhibiting the apoptosis.

RETRACTED

As shown in Figure 4, the results indicate that the increase of Bcl-2 expression and the decrease of Bax expression are involved in the antiapoptotic effect of salidroside. The next mission is to clarify how their expressions were influenced by salidroside. The upstream regulators of Bcl-2 mainly include p53, STAT3, NF-*κ*B p65, and PTEN. As shown in Figure 5, compared with H_2_O_2_ treatment, the expression of p53, p-STAT3, and p-p65 protein was significantly decreased by salidroside treatment in H_2_O_2_-stimulated H9C2 cells. Bcl-2 is one of STAT3 target genes, but the activation of STAT3 leads to the elevated expression of Bcl-2 and then promotes cell survival in oxidative stress. Translocation of NF-*κ*B p65 from cytoplasm into the nucleus can also bind to Bcl-2 promoter and regulate its expression. It indicates that the inhibition of NF-*κ*B p65 and STAT3 might not be involved in up-regulation of Bcl-2 by salidroside. PTEN is an inhibitor of Bcl-2; however, its expression was not changed by salidroside. On the contrast, the downregulation of p53 expression might be implicated in the antiapoptotic effect of salidroside. In our present study, the knockdown of p53 elevated the expression of Bcl-2 and decreased the expression of Bax in H_2_O_2_-stimulated H9C2 cells; furthermore, the overexpression of p53 exhibited the opposite result (Figure 6). Under physiological conditions, p53 plays an essential role in maintaining cardiac architecture and regulating the gene expressions associated with metabolism, mitochondrial biogenesis, cardiac architecture, and excitation-contraction coupling [24, 35], but the excessive expression of p53 is involved in the progress of heart failure. For example, the elevation of the p53 expression promotes the transition from compensated hypertrophy to decompensated heart failure undergoing pressure overload through p53-dependent apoptosis and antiangiogenesis [36–38]. The accumulated p53 can reduce the gene transcription of Bcl-2 through binding to the promoter of Bcl-2 [39, 40] and also directly interact with Bcl-2 to inhibit the complex formation between Bcl-2 and Bax [25]. In addition, p53 can also induce the gene transcription of Bax to decrease the ratio of Bcl-2/Bax [24, 25]. Therefore, the present results indicated that the inhibition of p53 is involved in the protective effects of salidroside against apoptosis induced by oxidative stress in H9C2 cells.

RETRACTED

## 5. Conclusion

In this study, salidroside inhibited the production of intracellular ROS to promote cell survival in H_2_O_2_-induced oxidative stress injury in H9C2 cells, which was associated with the restoration of the activity of antioxidant enzymes. Meanwhile, the apoptosis accompanied with oxidative stress was also reduced by salidroside through inhibiting p53 to elevate the expression of Bcl-2 and decrease the expression of Bax. Oxidative stress and excessive apoptosis are implicated in many heart diseases such as heart failure. Thus, salidroside is a promising natural compound in the treatment of myocardial diseases.

## Figures and Tables

**Figure 1:** Salidroside protected H9C2 cells against H_2_O_2_-induced injury. (a) H9C2 cells were treated with indicated concentration of salidroside for 24 h, and then cell viability was measured by MTT assay. (b) After incubation with H_2_O_2_ (0-800 *μ*M) for 4 h, the cell viability was measured by MTT assay. Experiments have been repeated five times. The values represent as means ± SD. ^∗^*p* < 0.05 vs. control. (c) H9C2 cells were treated with indicated concentration of salidroside for 24 h and then stimulated with or without H_2_O_2_ (400 *μ*M) for 4 h, and the cell viability was measured by MTT assay. (d) The level of ROS was detected using DCFH-DA. Experiments have been repeated four times. The values represent as means ± SD. ^∗^*p* < 0.05.

**Figure 2:** Salidroside protected H9C2 cells from H_2_O_2_-induced oxidative stress via enhancing antioxidant function. (a) The schematics of protective effect of salidroside against H_2_O_2_ induced damages. H9C2 cells were treated with indicated concentration of salidroside for 24 h and then stimulated with or without H_2_O_2_ (400 *μ*M) for 4 h. The activities of SOD (b), CAT (c), and the level of MDA (d) were detected. Experiments have been repeated five times. The values represent as means ± SD. ^∗^*p* < 0.05.

**Figure 3:** The effects of salidroside on the protein expressions of Bcl-2, Bax, and cleaved caspase-3 in H_2_O_2_-treated H9C2 cells. H9C2 cells were treated with salidroside (100 *μ*M) for 24 h and then stimulated with or without H_2_O_2_ (400 *μ*M) for 4 h. The protein expressions of Bcl-2, Bax, and caspase-3 were detected by western blot analysis. Experiments have been repeated five times. The values represent as means ± SD. ^∗^*p* < 0.05.

RETRACTED

**Figure 4:** Salidroside elevated the protein expression of Bcl-2 and inhibited cell apoptosis in H_2_O_2_-treated H9C2 cells. (a) H9C2 cells were transfected with siRNA targeting Bcl-2 (siBcl-2) or negative control (NC) using Lipofectamine3000 for 48 h and then harvested. H9C2 cells were transfected with siBcl-2 or NC for 24 h, and then the cells were treated with or without salidroside (Sal, 100 *μ*M) for 24 h and then stimulated with or without H_2_O_2_ (400 *μ*M) for another 4 h. (b) The protein expressions were detected by western blotting. (c) The morphological changes of apoptotic cells were observed by Hochest staining; (d) The apoptotic H9C2 cells were detected by flow cytometry. Experiments have been repeated four times. The values represent as means ± SD. ^∗^*p* < 0.05.

**Figure 5:** The effects of salidroside on the protein expressions of p53, p-STAT3, p-p65, and PTEN in H_2_O_2_-treated H9C2 cells. H9C2 cells were treated with or without salidroside (Sal, 100 *μ*M) for 24 h and then stimulated with or without H_2_O_2_ (400 *μ*M) for 4 h. The protein expressions were detected by western blotting. Experiments have been repeated four times. The values represent as means ± SD. ^∗^*p* < 0.05.

**Figure 6:** The decrease of Bcl-2 expression was involved in the increase of p53 expression in H_2_O_2_-treated H9C2 cells. (a) H9C2 cells were infected with Ad-GFP or Ad-p53 for 48 h. The protein expressions were detected by western blotting. (b) H9C2 cells were transfected with siRNA targeting p53 (sip53) or negative control (NC) using Lipofectamine3000 for 48 h. Western blotting was used to detect the knockdown efficacy of siRNA targeting p53. (c) H9C2 cells were transfected with sip53 or NC for 24 h, and then the cells were treated with or without H_2_O_2_ (400 *μ*M) for another 4 h. The protein expressions were detected by western blotting. Experiments have been repeated four times. The values represent as means ± SD. ^∗^*p* < 0.05.

## Data Availability

The data used to support the findings of this study are included within the article.
